# Inhibition of protein phosphatase 2A with a small molecule LB100 radiosensitizes nasopharyngeal carcinoma xenografts by inducing mitotic catastrophe and blocking DNA damage repair

This article has been retracted.

**DOI:** 10.18632/oncotarget.2258

**Published:** 2014-07-25

**Authors:** Peng Lv, Yue Wang, Jie Ma, Zheng Wang, Jing-Li Li, Christopher S. Hong, Zhengping Zhuang, Yi-Xin Zeng

**Affiliations:** ^1^ Cancer Institute and Hospital, Chinese Academy of Medical Sciences (CAMS),Beijing, People's Republic of China; ^2^ Beijing Neurosurgical Institute, Capital Medical University, Beijing, People's Republic of China; ^3^ Institute for Medical Device Standardization Administration, National Institutes for Food and Drug Control, Beijing, People's Republic of China; ^4^ Surgical Neurology Branch, National Institute of Neurological Disorders and Stroke, National Institutes of Health, Bethesda, MD,USA; ^5^ Department of Experimental Research, Sun Yat-sen University Cancer Center, Guangzhou, Guangdong, People's Republic of China; ^6^ State Key Laboratory of Oncology in Southern China, Guangzhou, Guangdong, People's Republic of China

**Keywords:** LB100, Radiosensitization, Protein phosphatase 2A, Nasopharyngeal Carcinoma

## Abstract

Nasopharyngeal carcinoma (NPC), while uncommon worldwide, is a major health problem in China. Although local radiation and surgery provide good control of NPC, better treatments that permit reductions in radiation dosing are needed. Inhibition of protein phosphatase 2A (PP2A), a ubiquitous multifunctional enzyme with critical roles in cell cycle regulation and DNA-damage response, reportedly sensitizes cancer cells to radiation and chemotherapy. We studied PP2A inhibition with LB100, a small molecule currently in a Phase I clinical trial, on radiosensitization of two human nasopharyngeal cell lines: CNE1, which is reportedly radioresistant, and CNE2. In both cell lines, LB100 exposure increased intracellular p-Plk1, TCTP, and Cdk1 and decreased p53, changes associated with cell cycle arrest, mitotic catastrophe and radio-inhibition of cell proliferation. Mice bearing subcutaneous xenografts of either cell line were administered 1.5 mg/kg LB100 daily for three days and a single dose of 20 Gy radiation (day 3), which produced marked and prolonged tumor mass regression (dose enhancement factors of 2.98 and 2.27 for CNE1 and CNE2 xenografts, respectively). Treatment with either LB100 or radiation alone only transiently inhibited xenograft growth. Our results support further exploration of PP2A inhibition as part of radiotherapy regimens for NPC and potentially other solid tumors.

## INTRODUCTION

NPC is the most common cancer of the nasopharynx, comprising 18 % of all cancers in China [1, 2], particularly in Guangdong province. Referred to as Cantonese Cancer because of its incidence of about 25 cases per 100,000 people in this region, NPC is much less common outside China, with less than 1 case per 100,000 in most populations [3]. Standard treatment is comprised of radiotherapy followed by surgical resection, resulting in high rates of local control, exceeding 90% [4]. However, improved treatments that in particular would allow for reduced radiation dosing are needed to both achieve long term control and reduce the high rates of radiation-induced temporal lobe necrosis often seen after radiation to the nasopharyngeal region [4, 5].

Protein phosphatase 2A (PP2A) is a ubiquitous and conserved serine/ threonine phosphatase that plays a role in many human pathological conditions, notably cancer [6, 7]. PP2A is a tumor suppressor and its function can be reduced by inactivating mutations of structural subunits or by up-regulation of cellular PP2A inhibitors [8-11]. However, PPA2 is also a negative regulator of cancer defense mechanisms activated in response to DNA damage by chemotherapy agents and radiotherapy [12]. Inhibition of PP2A has been reported to have anti-tumor activity against different human cancer cell types [13-17]. Sensitization of cancer cells to radiation and chemotherapy by PP2A inhibition is believed to occur via several mechanisms including sustained phosphorylation of p53, Akt, MDM2, Plk1, TCTP and Cdk1, which are associated with apoptosis, cell cycle deregulation, and inhibition of DNA repair [14, 18-22]. Thus, PP2A is a potential target for sensitization of tumors to both drugs and radiation [23].

LB100 is a water-soluble PP2A inhibitor currently in a phase I clinical trial [24]. In animal models of pheochromocytoma and sarcoma xenografts, LB100 treatment in combination with temozolomide or doxorubicin has been shown to significantly induce tumor regression without an apparent increase in systemic toxicity compared to either drug alone [14, 25]. In addition, a homolog of LB100, LB1.2, has been demonstrated to enhance the effectiveness of both temozolomide and doxorubicin against glioblastoma xenografts [13]. In the present study, we evaluated the effects of ionizing radiation (IR) therapy on PP2A activity and the ability of LB100 to enhance the therapeutic effects of radiation of against models of NPC.

## RESULTS

### LB100 demonstrates dose-dependent inhibition of NPC cells *in vitro*

CNE1 and CNE2 cells were exposed to different concentrations (1−200 μM) of LB100 or vehicle for 72 hours. MTT assays were used to measure the inhibition rates of cellular growth (Figure 1A, B). *In vitro*, LB100 showed little inhibitory activity at concentrations ≤ 5 μM but subsequently exhibited modest dose-dependent inhibition of CNE1 and CNE2 cell growth at higher concentrations. There were no significant differences in rates of apoptosis between CNE1 cells and CNE2 cells.

**Figure 1:** Effect of varying doses of LB100 on CNE1 and CNE2 cells *in vitro* Cultured CNE1 (A) and CNE2 (B) cells were treated with LB100 at the following concentrations: 0 (control), 1, 5, 10, 20, 50, 100, and 200 μM. Viable cells were counted at 24, 48, and 72 hours in triplicate by using MTT assay.

### LB100 exposure blocks radiation-induced increases in PP2A activity in NPC cells in vitro and in mouse xenograft models *in vivo*

PP2A has been shown to play a role in the ATM/ATR mediated activation of the G2/M cell cycle checkpoint, following radiation-induced DNA damage [20, 26]. We measured PP2A activity in CNE1 and CNE2 cells 6 hours after exposure to 8 Gy radiation *in vitro* and in CNE1 and CNE2 cell xenografts *in vivo* 6 hours after 20 Gy radiation, with and without prior exposure to LB100. Radiation *in vitro* was associated with increases of 260% and 210% in PP2A activity in CNE1 and CNE2 cells, respectively (Figure 2A). Radiation of xenografts *in vivo* was associated with increases in PP2A activity of 205% and 175% in CNE1 and CNE2 tumors, respectively (Figure 2B).

**Figure 2:** PP2A activity increases after radiation and is inhibited by LB100 *in vivo* and *in vitro* (A) PP2A activity of CNE1 and CNE2 cancer cells after treatment with 2.5 μM LB100 for 3 hours or with 8 Gy radiation after 6 hours. (B) PP2A activity of CNE1 and CNE2 subcutaneous xenografts treated with 1.5 mg/kg/day LB100 for 3 hours or with 20 Gy radiation after 6 hours. Data are the mean of triplicate samples (mean ± SE) and represent the percentage of PP2A activity as compared with control. Representative results shown are from three separate experiments (* ^Δ^ : VS control, p<0.05).

Exposure of both cell types to 2.5 μM LB100 alone for 3 hours reduced PP2A activity to 72% of control values in CNE1 and CNE2 cells (Figure 2A). In both cell line xenografts, intraperitoneal administration of a single dose of LB100 at 1.5 mg/kg also modestly reduced PP2A activity in both CNE1 and CNE2 xenograft tumors to 77% of controls (Figure 2B). However, when CNE1 and CNE2 cells were exposed to LB100 for 3 hours prior to 8 Gy radiation, the induction of PP2A was blocked, evidenced by a reduction in PP2A activity to 91% and 83% of control cells at 6 hours in CNE1 and CNE2 cells, respectively (Figure 2A). Similarly, when mice bearing CNE1 and CNE2 xenografts were treated with 1.5 mg/kg LB100 intraperitoneally for 3 hours prior to 20 Gy radiation, PP2A activity measured 6 hours after radiation was reduced to 87% and 81% of controls in CNE1 and CNE2 xenografts, respectively (Figure 2B).

### LB100 sensitizes NPC cells to the effects of radiation *in vitro*

Radiosensitization of NPC cells was determined via a clonogenic assay. CNE1 and CNE2 cells were exposed to 2.5 μM LB100 for 3 hours, which yielded cell survival fractions of 0.70 and 0.79, respectively. These results are within appropriate degrees of drug cytotoxicity for evaluation in combination with radiation. LB100 combined with radiation treatment strongly inhibited colony formation indicating significant radiosensitization, with dose enhancement factors (DEF) of 1.83 and 1.97 for CNE1 and CNE2, respectively (Figure 3A, B).

**Figure 3:** The effects of LB100 on radiosensitivity of CNE1 and CNE2 by clonogenic assay (A) and (B): Cells were assessed for clonogenic survival. Plots shown are representative of three separate experiments. Data in the legend are the mean DEF ± SE (n=3).

### LB100 radiosensitizes NPC xenografts

Mice bearing NPC subcutaneous xenografts were randomized to four treatment groups: vehicle alone, LB100 (1.5 mg/kg) alone, radiation (20 Gy) alone, and LB100 plus radiation. LB100 plus radiation inhibited CNE1 and CNE2 xenografts and prolonged survival (measured in days to a tumor volume ≥ 3000 mm^3^ at which point animals were euthanized) of the mice. The mean tumor weights and volumes of mice treated with radiation alone and with the combination of LB100 plus radiation were significantly less than those treated with vehicle or LB100 alone (Figure 4A-D). LB100 alone increased the time required for tumor volume doubling from 6.0 and 6.8 days in vehicle-treated animals to 6.4 and 8.1 days in CNE1 and CNE2 xenografts, respectively. Radiation alone slowed the rate of doubling to 9.2 and 10.6 days and decreased tumor weights to 61.7% and 65.2% of vehicle-treated animals for CNE1 and CNE2 xenografts, respectively. Lastly, LB100 in combination with radiation slowed the rate of tumor volume doubling to 27.7 and 26.7 days, which was associated with decreases in tumor weights of 87.6% and 88.0% relative to vehicle control in CNE1 and CNE2 xenografts, respectively (p<0.01; Figure 4E, F; Table 1). The DEF of LB100 for CNE1 and CNE2 subcutaneous xenografts were 2.98 and 2.27, respectively. The reportedly more radioresistant line, CNE1 [27, 28], was slightly more sensitive to enhancement of radiosensitivity by LB100 (Table 2). Survival times were significantly different between each treatment group and the control groups (p<0.05 for vehicle vs. LB100 and p<0.001 between all other groups; Figure 4G, H). The combination of LB100 and radiation was well tolerated and produced minimal (<10%) weight loss compared to controls, and the addition of LB100 caused no greater weight loss than radiation alone.

**Figure 4:** Radiosensitization of CNE1 and CNE2 xenografts by LB100 (A) and (B) Curve of CNE1 and CNE2 subcutaneous tumor volume treated with LB100 and radiotherapy at different time points. (C) and (D) Quantitative analysis of CNE1 and CNE2 xenograft weight after treatment with LB100 and radiation for 32 days (* : VS LB100 + radiation, p<0.05). (E) and (F) Statistically significant differences in tumor volume doubling are indicated versus PBS* and IR^Φ^. (G) and (H) Survival time after start of treatment of CNE1 and CNE2 xenografts. Mice in the combination LB100 plus radiation treatment group lived significantly longer than all other groups (p=0.001).

**Table 1:** Effects of treatment on tumor weights and tumor inhibition rate in model (mean ± SE, n=5)

Group	Number	Weight (g)		Tumor inhibition rate (%)	
		CNE1	CNE2	CNE1	CNE2
Control	5	3.48 ± 0.47^#^	4.06 ± 1.22^#^	-	-
LB100	5	3.05 ± 0.55^#^	4.08 ± 0.23^#^	12.30	-
Radiation	5	1.33 ± 0.76^#^^*^	1.41 ± 0.68^#^^*^	61.72	65.17
LB100+Radiation	5	0.43 ± 0.22	0.49 ± 0.28	87.64	87.98
F		35.38 32.31			
P	< 0.0001					

# VS LB100+Radiation;

* VS Control, p<0.05.

Note: Tumor inhibition rate (IR) = (1-tumor weight in experimental group/ tumor weight in vehicle control group) ×100%.

**Table 2:** Tumor diameter doubling time and growth delay in model (D) (mean ± SE, n=5)

Group	Diameter doubling time(D)		Growth delay(D)		Enhancement factor	
	CNE1	CNE2	CNE1	CNE2	CNE1	CNE2
Control	6.05 ± 0.31^#^	6.83 ± 0.37^#^		-	-	-
LB100	6.41 ± 0.73^#^	8.07 ± 0.21^#^	0.36	1.24	-	-
Radiation	15.22 ± 0.42^#^^*^	17.41 ± 0.63^#^^*^	9.17	10.58	-	-
LB100+Radiation	33.71 ± 0.55	33.57 ± 0.89	27.66	26.74	2.98	2.27
F					505.5	444.6
P	< 0.0001					

# VS LB100+Radiation;

* VS Control,p<0.01

Note: Enhancement factor(EF) = NGD/AGD Absolute growth delay (AGD) = TR-TC (defined as the time in days for tumors in the IR treatment group to grow doubling times in diameter minus the time in days for the tumors in the untreated control group to reach the same size). Normalized growth delay (NGD) = TL-TG (defined as the time in days for tumors in the combined treatment arm to grow doubling times in diameter minus the time in days for the tumors in the LB100 treated group to reach the same size).

These data demonstrate a synergistic effect between LB100 treatment and radiation, as evidenced by the significant abrogation of tumor growth delay and xenograft survival compared to radiation alone. As such, LB100 is a potent radiosensitizer *in vivo* in a NPC xenograft model.

### Radiosensitization induced by LB100 accumulates NPC cells in G2/M phase

Twenty-four hours after exposure to 2.5 μM LB100, CNE1 and CNE2 cells showed no significant difference in the distribution of cells in G0/G1 phase and S phase, compared to the control (Figure 5A). However, cells treated with LB100 and 8 Gy had a significantly higher proportion of cells in G2/M phase than control cells (Figure 5A-D). These data suggest that the radiosensitization induced by LB100 results from an accumulation of cells in G2/M phase rather than from drug-induced alterations in cell cycle distribution.

**Figure 5:** LB100 and IR induce cell cycle progression in CNE1 and CNE2 cells (A) PI staining and flow cytometry analyzed the G2/M rates of cell cycle in CNE1 and CNE2 cancer cells after treatment with 2.5 μM LB100 for 3 hours or 8 Gy radiation. (B) Quantification of data shown in panel A. (C) Cell cycle distribution after radiation and LB100 treatment. Data are the mean of triplicate samples (mean ± SE) and represent the percentage of surviving cells as compared with control. Representative results shown are from at least three separate experiments. (* ^Δ^ : VS control; ^Φ^ : VS CNE1, p<0.05).

### LB100 enhances apoptosis after radiation

To determine if induction of apoptosis contributes to radiosensitization *in vitro*, we measured apoptosis by flow cytometry 24 hours after treatment. The combination of 8 Gy and 2.5 μM LB100 produced significantly more apoptosis in both cell lines compared to LB100 alone (p=0.025) and to radiation alone (p=0.04) (Figure 6).

**Figure 6:** Cell apoptosis induced by LB100 and radiation (A) Annexin V-PI double staining and flow cytometry analyzed the apoptosis rates of CNE1 and CNE2 cancer cells, after treatment with 2.5 μM LB100 for 3 hours or 8 Gy radiation. (B) Quantification of data shown in panel A. Data are the mean of triplicate samples (mean ± SE) and represent the percentage of surviving cells as compared with control. Representative results shown are from at least three separate experiments. (* ^Δ^ : VS control; ^Φ^ : VS CNE1, p<0.05).

### LB100 activates CDK1 and enhances mitotic catastrophe in NPC cells

To explore the mechanisms responsible for LB100-mediated radiosensitization, we assessed changes in known PP2A substrates involved in the DNA damage response by Western blots. We measured the effects of LB100, radiation, and LB100 plus radiation on Plk1, Akt, p53, MDM2 and their downstream effectors, translationally controlled tumor protein (TCTP) and Cdk1 *in vitro*.

Exposure of CNE1 and CNE2 cells to LB100 for 6 hours resulted in the appearance of abnormal mitotic figures characteristic of mitotic catastrophe, a form of cell death distinct from apoptosis and cell senescence (Figure 8) [29, 30]. Induction of mitotic catastrophe by LB100 was associated with increased levels of phosphorylated Plk1 (p-Plk1), phosphorylated Akt (p-Akt1) and decreased levels of TCTP (Figure 7). TCTP is an abundant, highly conserved, multifunctional protein that binds to and stabilizes microtubules before and after mitosis and also exerts potent anti-apoptotic activity [31, 32]. Decreasing TCTP with antisense TCTP has been shown by others to enhance tumor reversion of v-src-transformed NIH 3T3 cells, and reduction of TCTP is suggested to be the mechanism by which high concentrations of certain anti-histamines and psychoactive drugs inhibit growth of a human lymphoma cell line [33].

**Figure 7:** Protein changes in CNE1 and CNE2 cells induced by LB100 and radiation Representative images of immunoblotting of p-Akt, total-Akt, p-Plk1, total-Plk1, TCTP, p-MDM2, total-MDM2, p53(Ser15), total-p53, p-Cdk1, total-Cdk1, γ-H2AX, total-H2AX, and β-actin in CNE1 and CNE2 cells treated with 1.5 mg/kg/day of LB100 for 3 hours, 20 Gy radiation at the dose of 600 cGy/min after 6 hours, and both treatments.

**Figure 8:** LB100 leads to persistent radiation-induced DNA damage (A) CNE1 and CNE2 cells were treated with 2.5 μM LB100 for 3 hours pre- and 24 hours post-radiation (8 Gy). At the end of drug exposure, cells were fixed and then subjected to immunofluorescence staining with DAPI and FITC for γ-H2AX. Representative images are shown. (B) Cells with more than 10 foci were scored as positive and plotted data are the mean ± SE of n=5-7 fields obtained from three separate experiments (*: VS control; ^Φ^ : VS IR, p<0.05).

LB100 exposure also was associated with an increase in phosphorylated MDM2 (p-MDM2), the primary regulator of p53 activity [34, 35], and a decrease in Ser15-phosphorylated p53 [p53(S15)] (Figure 7). An increase in MDM2 impairs p53-mediated arrest of the cell cycle allowing DNA replication and mitosis to proceed despite induced DNA damage [36]. p-Akt1 can stabilize MDM2 via phosphorylation and can also phosphorylate MDMX, which binds to and further stabilizes MDM2 [37].

p-Akt1 phosphorylation at Ser-308 indicates downstream activation of the phosphatidylinositol-3-kinase (PI3K) pathway, an event generally considered to be cell growth promoting [38]. Akt1 activation, however, may be anti- or pro-apoptotic depending on the context of cell signaling [39]. In the case of LB100 inhibition of PP2A, an increase in p-Akt1 activates Plk-1, a regulator of a mitotic checkpoint and of the activity of TCTP and Cdk1 [40, 41]. At the same time, increased p-Akt1 blocks cell cycle arrest mediated by p53 in response to DNA-damage [42].

Additionally, we found that LB100 alone and in combination with radiation were associated with an increase in Cdk1 activity via phosphorylation of Plk1 (Thr-210), ultimately resulting in persistent phosphorylation of Cdk1 at Tyr-15 [p-Cdk1(Y15)] and G2/M phase entry in response to DNA damage (Figure 7). Phosphorylation of Cdk1, a highly conserved serine/threonine kinase, is known to lead to cell cycle progression [43, 44].

Taken together, these data demonstrate a series of molecular changes in response to inhibition of PP2A by LB100, which likely result in blocking cell cycle arrest and inducing mitotic catastrophe via activation of Cdk1 and inhibition of TCTP.

### Effect of LB100 on repair of radiation-induced DNA double-strand breaks

To assess the effects of LB100 treatment on DNA damage and repair, we determined γ-H2AX levels, a measure of DNA double-strand breaks, at 6 hours in CNE1 and CNE2 cells by immunoblotting and immunofluorescence [18, 19, 45]. 2.5 μM LB100 alone caused no significant change in γ-H2AX levels. However, combined treatment with LB100 and radiation (8 Gy) or radiation alone was associated with similarly significant elevations in γ-H2AX expression in control and drug-treated CNE1 and CNE2 cells (Figures 7 and 8). Collectively, these data suggest that in NPC cells, LB100 interferes with cellular responses to DNA damage by preventing repair of radiation-induced DNA double-strand breaks, ultimately leading to persistent DNA damage and enhancement of radiation-induced cell killing.

## DISCUSSION

Our findings demonstrate that LB100, a small molecule inhibitor of PP2A, enhances the radiosensitivity of human NPC cells *in vitro* and *in vivo*. The potential for PP2A inhibition as an effective strategy for radiosensitization has been suggested previously [13, 20, 29, 46]. Earlier studies showed that the cyanobacterial toxin microcystin-LR, a PP1 and PP2A inhibitor, decreased repair of radiation-induced DNA damage in lymphocytes [47, 48]. In comparison, our results demonstrated higher DEF values when radiation was administered in conjunction with LB100. Furthermore, unlike previous studies involving LB100, we administered radiation as a single high dose rather than multiple low doses. Our data suggest a single potent dose of radiation may work well with LB100. Alternatively this effect could be also related to the biological entity of NPC or a unique genetic background in these NPC lines.

In the present study, radiosensitization of CNE1 and CNE2 cells by LB100 resulted from blocking cell cycle arrest and facilitating mitotic catastrophe rather than from an increase in apoptosis. LB100 exposure was associated with an increased percentage of cells in mitosis after radiation treatment. There are several possible explanations for this finding. One possibility is that PP2A inhibition results in abrogation of the G2/M checkpoint, allowing more cells to enter mitosis after radiation. An alternative possibility is that PP2A inhibition prevents cells from exiting mitosis. There is accumulating evidence that PP2A activity in association with B55α and B55δ regulatory phosphatase subunits is necessary for mitotic exit in mammalian cells [49, 50].

PP2A gene knockdown and protein inhibition by calyculin A are associated with ionizing radiation-induced phosphorylation of p53 at Ser46 and subsequent apoptosis in lymphocytes and Jurkat cells [22, 51, 52]. Our data indicate that in NPC cells inhibition of PP2A by LB100 triggers a chain of alterations in cancer cell signaling that accelerates inappropriate entry of cells into mitosis and, at the same time, impairs arrest of cell cycle at G1 and G2/M (Figure 9). In the face of radiotherapy-induced DNA damage and disordered cell replication, LB100 up-regulates Akt1, which has the potential to stimulate cell growth, and, at the same time, interferes with p53-mediated cell cycle arrest by stabilizing MDM2 [39]. An increase in p-Akt1 activates Plk1, interfering with the G2/M checkpoint [53, 54], up-regulates Cdk1 by dephosphorylation, and down-regulates TCTP by phosphorylation [30].

**Figure 9:** Schematic illustration of the potential mechanisms by which PP2A inhibition with LB100 enhances the effect of NPC radiotherapy

We also found that p-Plk1 phosphorylation of TCTP results in a marked reduction in TCTP abundance. Phosphorylation of TCTP decreases the stabilization of microtubules [31, 32], which may contribute to the development of mitotic catastrophe after exposure of cancer cells to LB100. Loss of TCTP expression during embryogenesis increases cell death [55], presumably by reduction of TCTP anti-apoptotic activity that is mediated by interference with Bax dimerization in the mitochondrial membrane [32]. Loss of TCTP induced by inhibition of PP2A may enhance cancer cell killing by causing persistent phosphorylation of γ-H2AX [18]. Our data show that inhibition of PP2A by LB100 is associated with only a slight increase in γ-H2AX levels. However, there was significantly increased γ-H2AX expression at 6 hours after radiation following LB100 suggesting that LB100 inhibits the repair of radiation-induced DNA damage in CNE1 and CNE2 cells. Extension of the *in vitro* data to an *in vivo* model confirmed that LB100 inhibits PP2A and prevents radiation-induced increases in PP2A activity whereas LB100 alone causes only a minor delay in tumor growth.

Wei et al recently reported that inhibition of PP2A sensitizes human pancreatic cancer cell lines *in vitro* and *in vivo* by inhibition of homologous recombination repair of DNA and activation of Cdc25c/Cdk1 signaling, suggesting that inhibition of PP2A is a potential target for enhancing local therapy in pancreatic cancer [56]. Our results indicate that LB100 is an effective and tolerable agent for sensitizing NPC cells to radiation in mouse models and provides additional support for preclinical exploration of the radiosensitizing properties of LB100 and other PP2A inhibitors. If the degree of radiosensitization seen in our studies of NPC in animal models can be achieved in humans without undue toxicities, the addition of LB100 to radiotherapy may increase the efficacy and lower the costs of NPC treatment. The results of a recently initiated Phase I trial will be instructive in the safety and tolerability of LB100 in humans.

## METERIALS AND METHODS

### Cell culture and drug solutions

Human nasopharyngeal carcinoma cell lines CNE1 and CNE2 were obtained from Sun Yat-sen University Cancer Center and grown in 1640 medium with 10% fetal bovine serum (FBS), penicillin and streptomycin. CNE1 cells are reported to be more radioresistant than CNE2 cells [57, 58].

Cell cultures were maintained in an atmosphere of 5% CO2/95% air at 37°C and tested free of Mycoplasma contamination. LB100, a water-soluble homolog of LB1.2 is a specific competitive small-molecule inhibitor of PP2A [13, 24]. LB100 was provided by Lixte Biotechnology Holdings Inc. (East Setauket, NY). It was stored at 1 mM in normal saline at -80°C.

### PP2A activity assay

At 80% confluence, cells were treated with LB100 (2.5 μM) or an equivalent volume of vehicle 3 hours prior to 8 Gy or sham radiation. Cells were washed three times in 0.9% saline. Tissue protein extraction reagent (T-PER) (Pierce Biotechnology, Rockford, IL) was added. 300 μg of cell lysate was assayed by Malachite Green Phosphatase assay for serine/threonine phosphatase activity (Ser/Thr phosphatase assay kit 1; Millipore, Billerica, MA). PP2A activity in CNE1 and CNE2 xenografts was assayed in the same conditions. *In vivo* LB100 dose was given at 1.5 mg/kg intraperitoneally daily for 3 days and radiation, 20 Gy at rate of 600 cGy/min, was given on day 3.

### Clonogenic survival assay

Cell cultures were trypsinized to generate single-cell suspensions and cells were seeded into 60mm dishes at cloning densities in duplicate or triplicate. After 24 hours, drug was added (2.5 μM, LB100). Cells were irradiated 3 hours later and the drug removed after 24 hours, followed by incubation at 37°C for 10 days. Colonies were stained with 0.2% crystal violet and the number of colonies containing at least 50 cells was determined. The surviving fractions were calculated and survival curves generated using the linear-quadratic equation after normalizing for cytotoxicity from LB100 treatment alone.

### Cell cycle analysis

Evaluation of cell cycle was performed by flow cytometry. Cells were exposed to LB100 (2.5μM) for 3 hours prior to administration of 8 Gy or sham radiation. Cells were trypsinized, fixed and stained per manufacturer's instructions with Cell Cycle Reagent, and analyzed on an EasyCyte Plus flow cytometer (Guava Technologies, Hayward, CA).

### Apoptosis assay

Apoptotic fraction was evaluated by flow cytometry using the Guava Nexin assay (Guava Technologies, Hayward, CA). Cells were exposed LB100 (2.5 μM) for 3 hours prior to administration of 8 Gy or sham radiation. Cells were trypsinized and stained per manufacturer's instructions with Nexin Reagent to assess annexin-V conjugated to phycoerythrin as a marker of cells in early apoptosis and 7-AAD as an indicator of late apoptosis (Guava Technologies). Analysis was performed on an EasyCyte Plus flow cytometer.

### γ-H2AX immunofluorescence assay

Immunofluorescent cytochemical staining for γoH2AX foci was performed by exposing cells grown on coverslips to LB100 (2.5 μM) for 3 hours prior to administration of 8 Gy or sham radiation. Cells were fixed with 4% paraformaldehyde, washed with PBS, permeabilized with 0.5% Triton X-100 in saline, blocked with 15% FBS in PBS, and incubated in blocking buffer containing primary antibody against γ-H2AX (Millipore) and then incubated with FITC-labeled goat anti-mouse IgG (Invitrogen, Carlsbad, CA). Nuclei were counterstained with DAPI (Sigma, St. Louis, MO). Cover slips were mounted with Beyotime anti-fade solution (Beyotime institute, Jiangsu, China) and γ-H2AX foci were imaged (40x objective) with a fluorescent microscope (BX51 Olympus microscope, Tokyo, Japan) and a Evolution^TM^ VF camera (Media Cybernetics, Rockville, MD).

### Immunoblotting

Whole cell and homogenized tissue lysates were prepared in cold RIPA buffer (50 mM Tris-HCl pH 7.5, 150 mM NaCl, 2 mM EDTA, 1% SDS, 0.2% Triton X-100 and 0.3% NP-40) supplemented with phosphatase and protease inhibitors (Roche, Basel, Switzerland) as previously described [59]. The protein concentration in each sample was measured by a colorimetric assay (ProteinAssay Kit; Bio-Rad Laboratories, Hercules, CA). Detection of protein bound primary antibodies was performed with a horseradish peroxidase conjugated secondary antibody specific to rabbit Ig and an enhanced chemiluminescence system. The following antibodies were used: PP2A, TCTP, Plk1, phospho-Plk1 (Thr20), phospho-Cdk1 (Tyr15), Cdk1 (Abcam, Cambridge, England), phospho-MDM2 (Ser166), phospho-Akt (Thr308), phospho-P53 (Ser15), Akt (Cell Signaling Technology, Danvers, MA), γ-H2AX, H2AX (Millipore), β-actin (Sigma).

### Animal experiments

BALB/c nude mice at 6-8 weeks of age were purchased from HFK Bio-technology Co. Ltd., Beijing, China. Each mouse weighed approximately 20 grams (half male and female). Animals were fed animal chow and water ad libitum and maintained on a 12-hour light/12-hour dark cycle. All animal experiments were carried out according to a protocol approved by the University Committee for Use and Care of Animals. Five million CNE1 and CNE2 cells in a 1:1 mixture of 10% FBS-1640 were injected subcutaneously into the right posterior limbs of BALB/c nude mice. When average tumor volume reached the size of approximately 120 mm^3^, the mice were randomized and the treatment was initiated. Animals were randomized into untreated controls, LB100, irradiation, and combination LB100 and irradiation. LB100 was administered daily Monday to Wednesday for 3 days, alone or in combination with radiation, at 1.5 mg/kg intraperitoneally. Radiation was administered at 20 Gy (600cGy/min) alone on day 3 or in combination 3 hours after LB100 treatment on day 3. Animals were restrained in lead jigs custom made by the Radiation Biology Branch of the Cancer Institute & Hospital, Chinese Academy of Medical Sciences. The growth of tumors (5 for each group) were measured five times per week and average tumor volume (TV) was calculated according to the equation: TV = (L× W^2^)/2, where L and W are the longer and shorter dimensions of the tumor, respectively. Animals were euthanized when tumors reached ≥ 3000 mm^3^. Survival was assessed by the Kaplan-Meier method with the day of injection assigned as day zero and a log-rank test used to compare groups.

### Ionizing Radiation

Ionizing radiation was carried out using a Varian-600CD linear accelerator (Varian, USA) at a dose rate of 600cGy/minute in the Department of Radiation Oncology of the Cancer Institute & Hospital, Chinese Academy of Medical Sciences. Dosimetry was carried out using an ionization chamber connected to an electrometer system that is directly traceable to a National Institute of Standards and Technology calibration. For tumor irradiation, animals were anesthetized with sodium pentobarbital and positioned such that the apex of each flank tumor was at the center of a 2.4 cm aperture in the secondary collimator, with the rest of the mouse shielded from radiation. The tissue-equivalent compensator was a 1 cm thick wax plate.

### Statistical analysis

*In vitro* studies were done in three independent experiments and the data are presented as mean ± SE. For *in vivo* tumor growth studies, log-rank tests were conducted to compare tumor volume doubling/tripling times between treatment arms. Time to tumor volume doubling/tripling was defined as the earliest day on which the tumor volume was at least twice/thrice as large as on the first day of treatment. A two-sided Student's t-test was used to compare sample means with a p value of <0.05 considered significant. All statistical analyses were carried out using GraphPad Prism 4 (San Diego, CA) and SigmaPlot software (Version 9.0, Systat Software Inc., San Jose, CA).
